The article "KLHDC8A Expression in Association with Macrophage Infiltration and Oxidative Stress Predicts Unfavorable Prognosis for Glioma" was retracted in 2023. Reasons: signs of a paper mill; suspected computer-generated content; unreliable results or conclusions; concerns about the data.

# KLHDC8A Expression in Association with Macrophage Infiltration and Oxidative Stress Predicts Unfavorable Prognosis for Glioma

**DOI:** 10.1155/2022/2694377

**Published:** 2022-09-19

**Authors:** Tong Cheng, Manyu Xu, Hui Zhang, Bing Lu, Xiaojing Zhang, Ziheng Wang, Jianfei Huang

**Affiliations:** Department of Clinical Biobank, Affiliated Hospital of Nantong University & Medical School of Nantong University, Jiangsu 226001, China

## Abstract

**Background:**

The tumor immune microenvironment (TME) is associated with cancer progression and immune escape. Although KLHDC8A has been reported in glioma *in vitro*, the expression and clinical significance of this gene in clinical samples are unknown.

**Methods:**

The Cancer Genome Atlas and Chinese Glioma Genome Atlas databases were used to evaluate the mRNA expression level of *KLHDC8A* and its significance in the glioma TME. Tissue microarray-based multiple immunohistochemical staining was conducted to determine KLHDC8A protein levels and characterize the immune signature of tumor-infiltrating immune cells in gliomas.

**Results:**

Tumor cells and tumor-associated macrophages expressed KLHDC8A. The expression of KLHDC8A was higher in glioma tissues than in normal brain tissues and was associated with patient clinical characteristics. Gliomas exhibited a high abundance of macrophages, neutrophils, regulatory T cells, and the immune checkpoint PD-L1, as well as high KLHDC8A expression. Cox regression analysis showed that KLHDC8A+CD68+ macrophages and KLHDC8A predicted unfavorable survival in patients with glioma. Finally, protein-protein interaction network analysis showed that the KLHDC8A expression was associated with hypoxia and oxidative stress.

**Conclusions:**

KLHDC8A is a potential marker for the clinical diagnosis of glioma. The immune characteristics of macrophages play a crucial role in predicting patients with glioma, providing a new avenue for targeted glioma therapy.

## 1. Introduction

Glioma is a tumor of the central neural system that affects the brain and spinal cord [1]. It comprises 81% of craniocerebral malignancies and is the most typical frequent primary tumor of the central nervous system [2]. According to the World Health Organization (WHO), gliomas are classified into four grades based on predicted clinical characteristics [3, 4]. The poorest five-year survival rate is for glioblastoma, while the highest relative survival rate is for pilocytic astrocytomas [5]. Furthermore, patients with glioma with IDH mutations have better survival [6, 7]. The prognosis for most patients with glioma remains poor, although survival rates for those undergoing concomitant chemotherapy and postoperative radiation therapy improve. Immunotherapy has long been recognized as a potential therapeutic strategy against cancer, and such new mechanisms may markedly improve the efficacy of immunotherapy for glioma.

The article "KLHDC8A Expression in Association with Macrophage Infiltration and Oxidative Stress Predicts Unfavorable Prognosis for Glioma" was retracted in 2023. Reasons: signs of a paper mill; suspected computer-generated content; unreliable results or conclusions; concerns about the data.

The brain tumor microenvironment (TME) is vital in primary and metastatic brain malignancies [8]. Tumor-infiltrating immune cells (TIICs) in the TME can accelerate tumor progression [9, 10]. Increasing evidence suggests that tumor-associated macrophages (TAMs) promote cell proliferation and invasion in glioma [11]. Importantly, TAM inhibition strongly blocks glioma formation [12]. TAMs, which are characterized by the expression of CD163, CD204, or CD206, support tumor growth [13]. Therefore, it is imperative to identify macrophage-related markers in the TME for developing targeted immunotherapies and identifying promising new therapeutic targets [14]. Simultaneously, hypoxia and radioresistance are closely associated with glioma. Moreover, oxidative stress, which is involved in central nervous system disorders, may lead to structural and functional disorders [15]. During oxidative stress, excessive production of reactive oxygen species (ROS) and reactive nitrogen species (RNS) can lead to neuronal dysfunction and death [16].

Based on bioinformatics approaches, KLHDC8A was screened as a hub gene by differential expression analysis. *KLHDC8A* encodes for Kelch domain-containing proteins that belong to the Kelch superfamily [17]. Several Kelch proteins play essential roles in many human diseases, including tumor and neurological diseases. The expression of Kelch proteins is upregulated in cancer [18–20]. Proteins belonging to the Kelch superfamily participate in extracellular interactions, cell migration, cell morphology, gene expression, and protein degradation [21, 22]. Overexpression of KLHDC8A drives the generation and development of glioma and the proliferation, migration, and invasion of glioma cells [23]. Additionally, the pathogenesis of glioma is considerably related to the abundance of immune components [24]. People with compromised immune systems are more likely to suffer from brain tumors [25–27]. However, the relationship between KLHDC8A expression and the glioma immune microenvironment has not been reported. Therefore, the role of KLHDC8A in the glioma TME deserves further investigation.

Using multiplex immunohistochemistry (mIHC) analysis and constructive tissue microarrays (TMAs), the current study assessed the expression of the KLHDC8A protein. The findings showed the role of KLHDC8A in the immunological milieu of gliomas by contrasting the expression of KLHDC8A with the abundance of TIICs and oxidative stress.

## 2. Methods

### 2.1. Patients and Tissue Samples

Transcriptome profiles and clinical information of 689 patients with glioma and 1152 healthy individuals were downloaded from The Cancer Genome Atlas (TCGA) (https://portal.gdc.cancer.gov/) and GETx databases, respectively. The Chinese Glioma Genome Atlas (CGGA) database (http://www.cgga.org.cn/index.jsp) was used to download microarray data of 301 patients with glioma, excluding missing information such as tumor grade (three cases), overall survival (sixteen cases), and age (two cases). Tissue samples were retrospectively collected from 231 patients (203 glioma tissues and 28 normal brain tissues) between 2012 and 2017 from the Clinical Biobank of Affiliated Hospital of Nantong University. In advance of surgery, there had been no radiotherapy, chemotherapy, immunotherapy, or other treatments. Ethics approval was obtained from the Affiliated Hospital of Nantong University.

The article "KLHDC8A Expression in Association with Macrophage Infiltration and Oxidative Stress Predicts Unfavorable Prognosis for Glioma" was retracted in 2023. Reasons: signs of a paper mill; suspected computer-generated content; unreliable results or conclusions; concerns about the data.

### 2.2. Immune Cell Infiltration Analysis

CIBERSORT is a computational algorithm for quantifying cell composition based on the expression profile of tissue genes [28]. The CIBERSORT algorithm was applied to estimate 22 distinct immune cell types [29]. Based on the mRNA expression of *KLHDC8A*, a high-expression group and a low-expression group were formed. To evaluate the relationship between KLHDC8A and TIICs, the median value of gene expression was set to 11.6.

### 2.3. Tissue Microarray and Immunohistochemical Staining

A tissue microarray (TMA) was constructed by the manual Tissue Microarrayer System Quick Ray (UNITMA, Seoul, Korea). TMA slides were prepared from surgically resected continuous specimens, fixed with formalin, and embedded in paraffin. A sample was represented as a core with a diameter of 2 millimeters on the TMA. The samples were dewaxed and hydrated using xylene (Changshi, China) and alcohol (ANNJET, China), respectively. Then, TMA slices were placed in sodium citrate buffer (Biosharp, China) (0.5 M, pH = 6.0) for antigen retrieval by microwave irradiation. TMA slides were then incubated with endogenous peroxidase (Maxim Biotechnologies, China) blocker for 20 min, followed by 5% Bovine serum albumin (BSA, biofroxx, China) blockade for 20 min to remove background noise. Slides were incubated with rabbit anti-PD-L1 primary antibody at 4°C overnight. Then, the sections were incubated with a reaction enhancer solution (Maxim Biotechnologies, China) for 30 min, followed by incubation with a secondary antibody (Maxim Biotechnologies, China). Then, TMA slides were stained using an EliVision Plus DAB Kit (Kit-0015; Maxim Biotechnologies, Fuzhou, China) following the manufacturer's instructions, and the nuclei were stained with hematoxylin (Yizhiyuan, China). Slides were imaged using the Vectra3-automated imaging software, and images were analyzed and scored using inForm4.1.0 (Perkin Elmer). The staining intensity was scored as follows: 0 (no staining); 1+ (weak staining); 2+ (moderate staining); or 3+ (intense staining). The final staining score was calculated by summing the proportion of cells stained at each intensity and the intensity score (0-300).

The article "KLHDC8A Expression in Association with Macrophage Infiltration and Oxidative Stress Predicts Unfavorable Prognosis for Glioma" was retracted in 2023. Reasons: signs of a paper mill; suspected computer-generated content; unreliable results or conclusions; concerns about the data.

### 2.4. Multiple Immunohistochemical Staining

An Opal 7-Color Manual IHC kit (PerkinElmer, NEL811001KT) was used to perform multiple immunohistochemical staining (mIHC) analysis. Formalin-fixed paraffin-embedded tissue sections were prepared by microwave heating in AR6 buffer (AR600, AKOYA). Slides were blocked with a blocking buffer (ARD1001EA, AKOYA) for 10 min. On the next day, the slides were rewarmed for 30 min and were incubated with the second antibody Opal™ polymer HRP Ms + Rb (ARH1001EA, Perkin Elmer) at room temperature for 10 min. Then, the nuclei were counterstained blue with DAPI (F6057, Sigma). The primary antibodies used in our study are listed in the supplementary materials (Supplementary Table S1).

Each sample was captured at a 20x magnification using the Vectra3-automated imaging software. The images were analyzed and scored using inForm4.1.0 (Perkin Elmer), and a threshold for positive or negative cells was set for each cell. The percentage of cells in each region was calculated and scored (0-100).

### 2.5. Protein-Protein Interaction Analysis

The proteins directly interacting in a network can be identified by protein-protein interaction (PPI) analyses. STRING is a search tool for identifying interacting genes [30]. Using the STRING tool, a protein-protein network that displays the genes interacting with KLHDC8A and associated immunological markers was constructed.

### 2.6. Statistical Analysis

Differences between two groups were analyzed using Student's *t-*test. Based on KLHDC8A expression and abundance of CD68+ macrophages, patients were categorized into high and low groups using 52 and 10.14 as cutoff points, derived from the X-tile software. Moreover, TIIC abundances and KLHDC8A expression were correlated using Spearman's correlation coefficients. Nomogram construction was performed using “rms” and “survival” packages in R. Descriptive statistics of the cohorts were determined using SPSS version 23.0. Data were also processed using the R software (v.4.1.1). Statistical significance was set at *P* < 0.05.

## 3. Results

### 3.1. Correlation between *KLHDC8A* mRNA Expression and TIIC Abundance in Gliomas

In this study, we analyzed a cohort of 689 glioma tissues and 5 adjacent tissues with available mRNA expression and clinical information in TCGA database. A total of 1152 normal tissues from the GTEx database were also included. Compared with that in normal tissues, KLHDC8A expression was elevated in glioma tissues (Figure 1(a)). Based on KLHDC8A expression, patients were categorized into high- and low-expression groups according to the cutoff value of 11.6. Shorter survival was independently correlated with *KLHDC8A* expression (Figure 1(b)). Additionally, the CIBERSORT algorithm was used to assess the relative abundance of 22 types of TIICs in each TCGA sample. The heatmap presented an integrated immune cellular landscape of gliomas (Figure 1(c)). Furthermore, KLHDC8A expression was significantly correlated with the abundance of M2 macrophages (Spearman, *r* = 0.184, *P* < 0.001), neutrophils (Spearman, *r* = 0.35, *P* < 0.001), and regulatory T cells Tregs (Spearman, *r* = 0.247, *P* < 0.001) (Figure 1(d)). These data suggested an association between KLHDC8A expression and the immune microenvironment of gliomas.

The article "KLHDC8A Expression in Association with Macrophage Infiltration and Oxidative Stress Predicts Unfavorable Prognosis for Glioma" was retracted in 2023. Reasons: signs of a paper mill; suspected computer-generated content; unreliable results or conclusions; concerns about the data.

### 3.2. Multiplex Immunohistochemistry Revealed the Protein Expression Level and Localization of KLHDC8A

Since mRNA expression levels are not always indicative of protein levels [31, 32], we performed mIHC to detect the expression of KLHDC8A. In agreement with TCGA results, the KLHDC8A protein was highly expressed in glioma tissues (Figure 2(a)). Immunofluorescence staining revealed that KLHDC8A was also expressed in CD68+ macrophages (Figure 2(b)). Additionally, glioma tissues were enriched in KLHDC8A+CD68+ macrophages compared to normal brain tissues (Figure 2(c)).

### 3.3. KLHDC8A in Cancer and Macrophages in Relation to TIICs

To further verify the correlations between KLHDC8A expression and TIIC abundance in the immune microenvironment of gliomas, we conducted mIHC (Figure 3(a)). There was an extensive infiltration of CD25+ Tregs, CD66b+ neutrophils, CD68+CD163+ M2 macrophages, and S100A4+ CAFs in the glioma microenvironment. However, the infiltration of CD3+CD4+ T cells and CD3+CD8+ T cells was low (Figure 3(b)). The expression of KLHDC8A and the infiltration of KLHDC8A+CD68+ macrophages were positively related to the abundance of Tregs, neutrophils, and M2 macrophages (Figure 3(c), Supplementary Table S2). However, no significant correlation was observed between the infiltration of KLHDC8A+CD68+ macrophages and CAFs.

### 3.4. Correlation between KLHDC8A Expression and Clinical Features of Glioma

The clinical information of 203 patients with glioma, including age, sex, tumor grade, IDH1 mutation, and histological classification, was collected from the Affiliated Hospital of Nantong University. KLHDC8A expression in cancer and abundance of CD68+ macrophages were divided into high- and low-expression groups. Next, we analyzed the relationship between KLHDC8A expression and clinicopathologic features. According to the results, KLHDC8A expression in macrophages and cancer cells was correlated with tumor grades (Table 1). Additionally, the infiltration of S100A4+ CAFs, CD25+ Tregs, CD66b+ neutrophils, CD68+CD163+ M2 macrophages, and S100A4+CD163+ cells was correlated with the clinical characteristics of patients with glioma (Figures 4(a) and 4(b)). The infiltration of CD25+ Tregs, CD68+CD163+ M2 macrophages, and S100A4+CD163+ was increased with high expression of KLHDC8A and high infiltration of KLHDC8A+CD68+ macrophages. High KLHDC8A expression was associated with enhanced infiltration in S100A4+ CAFs, but KLHDC8A+CD68+ macrophage infiltration was not substantially different. The infiltration of CD66b+ neutrophils increased as that of KLHDC8A+CD68+ macrophages increased; however, no significant association was observed between KLHDC8A+CD68+ macrophage infiltration and KLHDC8A expression (Figures 4(c) and 4(d)). Compared to WHO grades I and II, S100A4+ CAFs, CD25+ Tregs, CD68+CD163+ M2 macrophages, and S100A4+CD163+ cells had elevated infiltration in grade III and IV tumors (Figure 4(e)). Concurrently, the infiltration of CD66b+ neutrophils did not significantly differ across tumor grades.

The article "KLHDC8A Expression in Association with Macrophage Infiltration and Oxidative Stress Predicts Unfavorable Prognosis for Glioma" was retracted in 2023. Reasons: signs of a paper mill; suspected computer-generated content; unreliable results or conclusions; concerns about the data.

### 3.5. High KLHDC8A and KLHDC8A+CD68+ Expression Predicted Unfavorable Prognosis in Glioma

A cohort of 280 patients with glioma from the CGGA database was included to further investigate the clinical outcome of KLHDC8A expression and TIIC abundance in patients with glioma using the Cox regression analysis. Prognostic factors associated with gliomas were KLHDC8A, age, IDH1, CD163, S100A4, and tumor grade (Figure 5(a)). Our findings demonstrated that KLHDC8A, KLHDC8A+CD68+ macrophages, age, sex, IDH1 mutations, and tumor grade were independent prognostic indicators for gliomas (Figure 5(b), Table 2). In contrast, CD25+ Tregs, CD66b+ neutrophils, CD68+CD163+ M2 macrophages, and S100A4+CD163+ cells were not related to clinical outcomes in patients with glioma. Furthermore, patients with high KLHDC8A expression had poorer survival outcomes than those with low KLHDC8A expression (Figure 5(c)). High expression of KLHDC8A in macrophages also contributed to the short overall survival (OS) of patients with glioma (Figure 5(d)). Simultaneously, patients with high tumor grades had an unfavorable prognosis (Figure 5(e)). Cox regression analysis was performed to investigate the predictive effects of KLHDC8A, KLHDC8A/CD68+ macrophages, sex, age, and tumor grade on the survival time of patients with glioma. A nomogram was constructed to indicate the 1-, 3-, and 5-year survival rates of patients with glioma in TCGA database and our trial cohort (Figures 5(f) and 5(g)).

The article "KLHDC8A Expression in Association with Macrophage Infiltration and Oxidative Stress Predicts Unfavorable Prognosis for Glioma" was retracted in 2023. Reasons: signs of a paper mill; suspected computer-generated content; unreliable results or conclusions; concerns about the data.

### 3.6. Biological Processes Enriched in KLHDC8A

Since PD-L1 plays an important role in the immunosuppression of gliomas, we further explored the association between the expression of KLHDC8A and that of PD-L1. We evaluated the relationship between KLHDC8A expression and multiple immune checkpoint molecules and found a significant difference between the expression of KLHDC8A and that of PD-L1 (Figure 6(a)).

Additionally, we performed IHC to evaluate the expression of PD-L1 in patients with glioma (Figure 6(b)) and found that the expression of KLHDC8A was significantly and positively correlated with that of PD-L1 (Figures 6(c) and 6(d)).

The STRING tool was used to develop a PPI network consisting of KLHDC8A, DEAF1, SOX2, S100A4, SLC16A4, MCTS1, CD68, HIF1A, ZEB1, SNAI1, CD163, and CD274. DEAF1, an essential regulator of innate immune responses [33], maintains immune cell functions by regulating the transcription of antigen-encoding genes in lymph node stromal cells [34]. However, it is still worth exploring whether the interaction between KLHDC8A and DEAF1 proteins can drive immune cells to affect glioma progression. MCT1, a lactate export protein, is mainly upregulated during hypoxia in glioma cells [35]. Simultaneously, hypoxia can induce epithelial-mesenchymal transformation (EMT) during glioma progression [36]. Hypoxia-induced EMT is usually regulated by EMT transcriptional regulators, including Snail, Twist1, and ZEB1 [37]. During EMT, tumor cells induce the release of chemokines from macrophages to promote interactions between TAMs and tumor cells to alter TAM phenotypes. The results showed that KLHDC8A expression was related to the expression of DEAF1, HIF1A, and MCTS1 (MCT1) (Figures 6(f)–6(h)). Additionally, we explored the association of KLHDC8A expression with ROS and RNS production. The results revealed that KLHDC8A was negatively correlated with ROS (ROS1) production, but it was significantly and positively correlated with RNS (FAM20C) production (Figures 6(i) and 6(j)).

## 4. Discussion

In this study, we performed bioinformatics analysis and mIHC staining to explore the relevance of KLHDC8A expression in the glioma immune microenvironment and its association with oxidative stress. The immunological microenvironment is important for the development of glioma, one of the most immunosuppressive solid tumors.

Macrophages are thought to contribute to tumor growth and progression and promote tumor cell survival, proliferation, and dissemination [11, 38]. Macrophages are an essential component of immune invasion in the glioma tumor microenvironment [39]. M2 macrophages can promote the progression and growth of glioma [40]. Upregulation of KLHDC8A contributes to the proliferation, migration, and invasiveness of glioma cells [23]. In this study, the significant association between KLHDC8A and the TME is worthy of further exploration. In this study, we used bioinformatics analysis and confirmed that KLHDC8A expression was closely related to glioma immune characteristics and oxidative stress.

The article "KLHDC8A Expression in Association with Macrophage Infiltration and Oxidative Stress Predicts Unfavorable Prognosis for Glioma" was retracted in 2023. Reasons: signs of a paper mill; suspected computer-generated content; unreliable results or conclusions; concerns about the data.

Our study indicated that KLHDC8A expression was correlated with CD68+, S100A4+, CD68+CD163+, and S100A4+CD163+ macrophage infiltration to varying degrees, and KLHDC8A was expressed on CD68+ macrophages. Furthermore, patients with high levels of macrophage infiltration of CD68+, CD163+, CD68+CD163+, and S100A4+CD163+ had shorter survival than those with low levels of macrophage infiltration. CD163+ TAMs promote tumor progression and affect prognosis [41]. Our results supported this and prompted the issue of whether the tumor-promoting activity of KLHDC8A may affect macrophage infiltration. Our findings are supported by this conclusion, and we also posed the issue of whether the tumor-promoting activity of KLHDC8A influences macrophage infiltration.

In addition to CD68+CD163+ M2 macrophages, we identified S100A4+CD163+ and KLHDC8A+CD68+ macrophage subsets. S100A4 enhanced the M2-like polarization of tumor macrophages [42]. Simultaneously, patients with high KLHDC8A+CD68+ macrophage infiltration had shorter survival than those with low KLHDC8A+CD68+ macrophage infiltration. Therefore, we identified two specific macrophage subgroups that are positively correlated with KLHDC8A expression and affect the prognosis of gliomas. Despite these results, more research is needed to determine if KLHDC8A may affect the development of glioma via a signaling route that affects macrophage infiltration.

Using the STRING database, we discovered that KLHDC8A interacts with MCTS1 and DEAF1 proteins. MCT1 and MCT4 have been shown to induce hypoxia and promote glioma cell proliferation and invasion in both *in vivo* and *in vitro* glioma models [35]. Moreover, the number of activated macrophages and rate of glycolysis were reduced after MCT4 knockdown [43]. These results suggest that KLHDC8A may affect glioma progression by targeting MCT1 to regulate macrophage phenotypes. DEAF1 is involved in the innate immune response *in vivo* [44]. As a critical inducer of EMT in cancer cells, ZEB1 can drive EMT in cancer cells to promote tumor progression [45]. Moreover, ZEB1 was upregulated in glioma, and its tumor-promoting function in tumor-associated macrophages was maintained [46]. However, whether KLHDC8A can drive glioma progression through ZEB1 and macrophage interactions needs to be explored. Blocking PD1 and PD-L1 interactions *in vivo* increased TAM phagocytosis and reduced tumor growth [47]. This result suggests that PD-1-PD-L1 therapy exerts its effect through macrophages, thereby making it suitable for clinical treatment. Oxidative stress enhances macrophage infiltration in glioma cells [48]. Increased ROS and RNS can induce oxidative stress [49]. The results of our analysis showed that KLHDC8A and RNS were significantly and positively correlated. We speculate that elevated RNS levels induce KLHDC8A expression, accelerating the progression of gliomas.

The article "KLHDC8A Expression in Association with Macrophage Infiltration and Oxidative Stress Predicts Unfavorable Prognosis for Glioma" was retracted in 2023. Reasons: signs of a paper mill; suspected computer-generated content; unreliable results or conclusions; concerns about the data.

There are several limitations to this study. First, the sample size was small; therefore, conclusions drawn from existing studies must be cautioned. This is a retrospective study. Our utilization of TMA allows us to study a large number of samples simultaneously, but due to the small core size, sample bias (including tumor heterogeneity) may be higher than in studies of whole sections. Our results do not necessarily imply that the infiltration of KLHDC8A+CD68+ macrophages detrimentally affects the prognosis of patients with glioma. We did not explore the interaction mechanism between KLHDC8A and immune cells in the immune microenvironment. Further *in vitro* and *in vivo* experimental evidence is needed to validate the findings of this study. Recently, immunotherapy has emerged as a novel and attractive therapeutic strategy against glioma. Nevertheless, the efficacy of immunotherapy is limited by glioma-induced immunosuppression. Therefore, the strategic targeting of cells in the immunosuppressive glioma microenvironment is an attractive alternative therapeutic approach.

In our study, global expression analysis revealed that KLHDC8A was upregulated in gliomas and associated with a poor prognosis. We highlighted the link between tumor-associated macrophages and KLHDC8A expression. We hypothesized that KLHDC8A might be a promising therapeutic target for gliomas.

## 5. Conclusion

KLHDC8A is a promising indicator for the clinical diagnosis of glioma. The immune characteristics of macrophages play a crucial role in predicting the prognosis of patients with glioma, providing a novel strategy for the targeted therapy of gliomas.

## Figures and Tables

**Figure 1:** *KLHDC8A* mRNA expression in gliomas. (a) *KLHDC8A* mRNA expression in normal and tumor tissues. (b) Patients with high *KLHDC8A* expression had a poor prognosis. (c) The heatmap represents the proportions of 22 distinct immune cell types. (d) KLHDC8A expression was correlated with tumor-infiltrating immune cell (TIIC) abundance in The Cancer Genome Atlas (TCGA) database.

The article "KLHDC8A Expression in Association with Macrophage Infiltration and Oxidative Stress Predicts Unfavorable Prognosis for Glioma" was retracted in 2023. Reasons: signs of a paper mill; suspected computer-generated content; unreliable results or conclusions; concerns about the data.

**Figure 2:** The protein expression level and localization of KLHDC8A. (a) KLHDC8A protein expression in glioma tissues. (b) Fluorescence-based multiplex immunohistochemistry revealed differences in the expression of the KLHDC8A protein between normal and tumor tissues. (c) The infiltration of KLHDC8A+CD68+ macrophages in the glioma microenvironment.

**Figure 3:** Correlation between KLHDC8A expression in cancer and macrophages and the abundance of tumor-infiltrating immune cells (TIICs). (a) Representative multiplex immunofluorescence staining images. (b) The infiltration levels of TIICs in gliomas. (c) KlHDC8A expression was related to TIIC abundance.

**Figure 4:** The relationship between KLHDC8A expression and the clinical features of glioma. (a, b) The heatmap shows the relationship between macrophage infiltration and clinical features in patients with glioma. (c, d) The expression of KLHDC8A was correlated with the abundance of tumor-infiltrating immune cells (TIICs). (e) Tumor grades were correlated with the abundance of TIICs.

**Figure 5:** High KLHDC8A and KLHDC8A+CD68+ expressions are independent prognostic factors for gliomas. (a) A forest plot revealed the effect of tumor microenvironment- (TME-) related features and KLHDC8A expression on overall survival (OS) in The Cancer Genome Atlas (TCGA) database. (b) A forest plot revealed the effect of TME-related features and KLHDC8A on OS in our cohort. (c) Kaplan–Meier curves of KLHDC8A high- and low-expression groups in our cohort. (d) Kaplan–Meier plot indicating the association of the abundance of KLHDC8A+CD68+ macrophages and OS. (e) Tumor grades were associated with patient survival. (f, g) Nomograms were constructed to evaluate the prognostic significance of immune features in TCGA database and our study cohort.

**Figure 6:** Exploration of biological processes associated with KLHDC8A. (a) Expression of different immune checkpoint molecules in the high and low KLHDC8A expression groups. (b) The representative immunohistochemistry (IHC) images of PD-L1 expression. (c, d) PD-L1 expression was positively correlated with KLHDC8A expression. (e) Construction of protein-protein interaction network. (f–h) KLHDC8A expression was correlated with DEAF1, HIF1A, and MCTS1 (MCT1). (i, j) KLHDC8A expression was correlated with the production of reactive oxygen species (ROS) (ROS1) and reactive nitrogen species (RNS) (FAM20C).

**Table 1:** Relationship between KLHDC8A expression and clinicopathological features.

Characteristic	KLHDC8A					KLHDC8A/CD68+				
	*n*	Low expression (%)	High expression (%)	Pearson *χ*^2^	*P*	*n*	Low expression (%)	High expression (%)	Pearson *χ*^2^	*P*
Total	203	126 (62.07)	77 (37.93)			203	41 (20.20)	162 (79.80)		
Sex				0.482	0.487				0.006	0.936
Male	115	69 (60.00)	46 (40.00)			88	18 (20.45)	70 (79.55)		
Female	88	57 (64.77)	31 (35.23)			115	70 (59.83)	47 (40.17)		
Age				0.996	0.318				0.404	0.525
≤60	130	84 (64.62)	46 (35.38)			130	28 (21.54)	102 (78.46)		
>60	73	42 (57.53)	31 (42.47)			73	13 (17.81)	60 (82.19)		
Histological classification				6.853	0.144				5.339	0.254
a (AA, AG, AOA, AGG, and PA)	35	28 (80.00)	7 (20.00)			35	11 (31.43)	24 (68.57)		
b (A)	84	50 (59.52)	34 (40.48)			84	17 (20.24)	67 (79.76)		
c (GBM)	50	28 (56.00)	22 (44.00)			50	9 (18.00)	41 (82.00)		
d (MG)	31	19 (61.29)	12 (38.71)			31	3 (9.68)	28 (90.32)		
e (DA and PPXA)	3	1 (33.33)	2 (66.66)			8	1 (33.33)	2 (66.66)		
IDH1				0.521	0.470				0.849	0.357
IDH1+	91	54 (59.34)	37 (40.66)				21 (23.08)	70 (76.92)		
IDH1-	112	72 (64.29)	40 (35.71)				20 (17.86)	92 (82.14)		
Grade				15.248	<0.001∗				6.257	0.044∗
I+II	42	34 (80.95)	8 (19.05)			42	13 (30.95)	29 (69.05)		
III	48	35 (72.92)	13 (27.08)			48	12 (25.00)	36 (75.00)		
IV	113	57 (50.44)	56 (49.56)			113	16 (14.16)	97 (85.84)		

^∗^ *P* < 0.05. a: anaplastic astrocytoma, glioma, ganglioglioma, oligoastrocytoma, oligodendroglioma, pilocytic astrocytoma, and pilomyxoid astrocytoma. b: astrocytoma. c: glioblastoma. d: mixed glioma. e: diffuse astrocytoma and pleomorphic xanthoastrocytoma.

The article "KLHDC8A Expression in Association with Macrophage Infiltration and Oxidative Stress Predicts Unfavorable Prognosis for Glioma" was retracted in 2023. Reasons: signs of a paper mill; suspected computer-generated content; unreliable results or conclusions; concerns about the data.

**Table 2:** Univariate and multivariable analyses of prognostic factors for 5-year survival in patients with glioma.

	Univariate analysis				Multivariate analysis			
	HR	*P* > |*z*|	95% CI		HR	*P* > |*z*|	95% CI	
KLHDC8A expression	3.787	<0.001^∗^	2.684	5.344	3.028	<0.001^∗^	2.001	4.581
KLHDC8A+CD68+ expression	2.271	0.001^∗^	1.430	3.606	1.822	0.022^∗^	1.090	3.044
Sex								
Male vs. female	1.461	0.024^∗^	1.052	2.030	1.701	0.004^∗^	1.188	2.433
Age (y)								
≤60 vs. >60	2.098	<0.001^∗^	1.514	2.907	1.687	0.007^∗^	1.151	2.472
Histological classification								
a (AA, AG, AOA, AGG, and PA) vs. b (A) vs. c (GBM) vs. d (MG) vs. e (DA and PPXA)	1.271	0.001^∗^	1.097	1.472	1.027	0.788	0.846	1.247
IDH1								
IDH1+ vs. IDH1-	0.660	0.011^∗^	0.479	0.910	0.653	0.018^∗^	0.459	0.928
S100A4	1.286	0.125	0.932	1.775				
CD25	1.410	0.046^∗^	1.006	1.976	0.386	0.846	0.579	1.235
Cd66b	1.289	0.133	0.925	1.795				
CD68+CD163+	2.170	<0.001^∗^	1.560	3.019	1.093	0.723	0.669	1.785
S100A4+CD163+	1.728	0.001^∗^	1.247	2.393	0.774	0.267	0.493	1.216
Grade								
I vs. II vs. III vs. IV	2.284	<0.001^∗^	1.803	2.893	1.716	<0.001^∗^	1.284	2.294

^∗^ *P* < 0.05. a: anaplastic astrocytoma, anaplastic glioma and anaplastic ganglioglioma. b: anaplastic oligoastrocytoma, astrocytoma, diffuse astrocytoma, and oligodendroglioma. c: glioblastoma. d: mixed glioma.

The article "KLHDC8A Expression in Association with Macrophage Infiltration and Oxidative Stress Predicts Unfavorable Prognosis for Glioma" was retracted in 2023. Reasons: signs of a paper mill; suspected computer-generated content; unreliable results or conclusions; concerns about the data.

## Data Availability

Data in support of this study are available from the corresponding author upon reasonable request.

## Supplementary Materials

Supplementary 1 The primary antibodies used in our study are listed in the supplementary materials (Supplementary Table S1).

Supplementary 2 The expression of KLHDC8A and the infiltration of KLHDC8A+CD68+ macrophages were positively correlated with the abundance of Tregs, neutrophils, and M2 macrophages.
